# Ecofriendly Synthesis of Silver Nanoparticles Using *Ananas comosus* Fruit Peels: Anticancer and Antimicrobial Activities

**DOI:** 10.1155/2021/2058149

**Published:** 2021-11-30

**Authors:** Ayşe Baran, Cumali Keskin, Mehmet Fırat Baran, Irada Huseynova, Rovshan Khalilov, Aziz Eftekhari, Sevgi Irtegun-Kandemir, Deniz Evrim Kavak

**Affiliations:** ^1^Department of Biology, Graduate Education Institute, Mardin Artuklu University, Mardin, Turkey; ^2^Department of Medical Services and Techniques, Vocational Higher School of Healthcare Studies, Mardin Artuklu University, Mardin, Turkey; ^3^Joint Ukrainian-Azerbaijan International Research and Education Center of Nanobiotechnology and Functional Nanosystems, Drohobych Ukraine & Baku, Azerbaijan; ^4^Institute of Molecular Biology & Biotechnologies, Azerbaijan National Academy of Sciences, 11 Izzat Nabiyev, Baku 1073, Azerbaijan; ^5^Department of Biophysics and Biochemistry, Baku State University, Baku, Azerbaijan; ^6^Institute of Radiation Problems, National Academy of Sciences of Azerbaijan, Baku, Azerbaijan; ^7^Toxicology and Pharmacology Department, Maragheh University of Medical Sciences, Maragheh, Iran; ^8^Drug Applied Research Center, Tabriz University of Medical Sciences, Tabriz 51664, Iran; ^9^Department of Medical Biology, Faculty of Medicine, Dicle University, Diyarbakir 21280, Turkey; ^10^Dicle University Science and Technology Research Centre, Dicle University, Diyarbakir 21280, Turkey

## Abstract

Metallic nanoparticles are valuable materials and have a range of uses. Nanoparticles synthesized from plant wastes by environment-friendly methods have attracted the attention of researchers in recent years. Also, the advantages of biological resources and synthesis methods are attracting attention. In this study, silver nanoparticles were synthesized from *Ananas comosus* fruit peels using ecofriendly method steps. The characterization of the particles obtained was determined by using a UV-visible spectrophotometer (UV-Vis.), Fourier transform infrared spectroscopy (FTIR), X-ray diffraction diffractometer (XRD), Fourier scanning electron microscope (FESEM), and transmission electron microscopy (TEM). The nanoparticles showed maximum absorbance at 463 nm, measuring 11.61 in crystal nanosize, and presented spherical in appearance. An antimicrobial activity test was determined with the minimum inhibition concentration (MIC) method. The nanoparticles showed promising inhibitory activity on the Gram-positive and Gram-negative pathogen microorganisms (*Escherichia coli* ATCC25922, *Staphylococcus aureus* ATCC29213, *Bacillus subtilis* ATCC11774, *Pseudomonas aeruginosa* ATCC27833 bacteria, and *Candida albicans* yeast) at low concentrations. The cytotoxic and growth inhibitory effects of silver nanoparticles on different cancer cell lines were examined via the MTT assay.

## 1. Introduction

Nanomaterials synthesized by different methods, produced with metallic nanoparticles, are very valuable products that can be used in many areas. Nanoparticles show biological, optical, magnetic, and catalysis properties depending on their shape and size [1]. Some features of nanoparticles (NPs) make them superior. Having a large surface area and being resistant to high temperatures are some of these. With these features, they can be used in many fields such as material science, pharmaceutics, and electronics [1].

Physical, chemical, and biological methods are used to synthesize nanoparticles [2]. Physical and chemical methods have certain disadvantages compared to biological methods. The presence of toxic chemicals in the synthesis stages and the difficulty of controlling these steps also bring along problems such as high energy requirements and increased costs. In that aspect, biological methods are more advantageous [3].

For nearly 5000 years, ancient civilizations used silver materials while consuming foods and beverages or storing them for a long time [4]. Especially for their antimicrobial effects [5], silver nanoparticles (AgNPs) are widely used in anticancer agents [6], cosmetics [7], the food industry [8], electronics, catalysis [9], and bioremediation [10] applications such as dye removal. There are many biological sources to synthesize these particles. Bacteria [11], algae [12], fungi [13], yeasts [14], and plants [2] are among these. Using plants offers several advantages over other biological resources. Factors such as the ease of application, no risk of pathogenicity, and lack of problems including production conditions are some of these. In the synthesis of AgNPs with plant sources, the root [15], peel [16], fruit [17], leaf [18], and flower [19] parts or the whole plant can be used [20].

Cancer, with its different types and difficult treatment process that is often insufficient, is a tough disease to cope with, in today's world [21]. A lot of research is being carried out to develop new treatment methods every day [22–24]. AgNPs can contribute to this process, in finding new and effective methods. There are some studies on the use of AgNPs as anticancer agents [22, 23]. The use of AgNPs as antimicrobial and anticancer agents has been revealed as a result of many studies [23, 24]. AgNPs obtained from plant sources exhibit a biocompatible structure which provides great convenience for medical applications [6, 12].

Antibiotic resistance of microorganisms poses a serious problem. Thousands of people succumb to these microorganisms and die due to hospital pathogens being resistant to the antibiotics used [11]. Studies have shown that AgNPs can, at this point, contribute to the search for antimicrobial agents against pathogenic microorganisms [5, 11]. This study aimed to synthesize AgNPs from waste *Ananas comosus* fruit peels economically and easily via an ecofriendly method that does not involve toxic chemicals, characterize them, and examine their anticancer and antibacterial activities.

## 2. Materials and Methods

### 2.1. Equipment and Chemicals

The AgNPs were characterized by using the UV-visible spectrophotometer (Perkin Elmer One, Waltham, Massachusetts, United States), Fourier transform infrared spectroscopy (FTIR, Perkin Elmer Spectrum One, Waltham, Massachusetts, United States), X-ray diffractometer (XRD, RadB-DMAX II computer-controlled), Fourier scanning electron microscope (FESEM, Quanta FEG 250), transmission electron microscope (TEM, Jeol Jem, 1010 Akishima, Tokyo), and energy dispersive X-ray diffraction (EDX, RadB-DMAX-ray diffractometer). A high-speed OHAUS FC 5706 model centrifuge (10.000 rpm, Parsippany, New Jersey, United States.) was used to precipitate the nanoparticles. Silver nitrate solution (2.5% (w/v) AgNO3 in H2O) and standard antibiotics (vancomycin, colistin, and fluconazole) were commercially purchased (Sigma-Aldrich, Saint Louis, MO, United States).

### 2.2. Preparation of Plant Extract and Stock Solution

The peels of *Ananas comosus* fruits were cut and removed. After washing with tap water several times followed by distilled water, the peels were dried at room temperature. These dried peels were cut into smaller pieces and prepared to weigh. 200 grams of the dried fruit peels was weighed and left to boil in 500 mL of distilled water, half covered. From the moment it started boiling, we waited for about 15 minutes and left it to cool fully covered. First, coarse filter paper and, subsequently, a filtering process with Whatman 0.1 mm filter paper were used. The extract was stored at + 4°C for use in the synthesis phase. A solution of 10 mM (millimolar) concentration was prepared from the solid AgNO_3_.

### 2.3. Synthesis and Characterization of AgNPs

The prepared 500 mL plant extract and 10 mM solution were mixed in a 1000 ml glass flask at room temperature by using a magnetic stirrer. The solution was observed for color changes.

Related to color changes, samples were periodically taken (30, 45, 60, 90, 120 min) and measurements were made with a UV-Vis spectrophotometer to determine the formation and presence of AgNPs. FTIR device frequencies were used for determining the functional groups responsible for the reduction. After the reaction, the dark liquid sample was centrifuged at 10.000 rpm and the precipitate was dried for other characterization processes. Crystal nanosize and structure were evaluated with XRD data. The FESEM, TEM, and EDX data were used to determine morphological structure and element composition.

### 2.4. Antimicrobial Assay

Microorganisms were provided by the Microbiology Laboratory of İnönü University's Medical Faculty Hospital (*Staphylococcus aureus* American Type Culture Collection (ATCC) 29213 and *Escherichia coli* ATCC25922 strains and *Candida albicans* yeast) and the Microbiology Research Laboratory of Artuklu University (*Bacillus subtilis* ATCC 11774 and *Pseudomonas aeruginosa* ATCC27833).

Microorganism suspensions were prepared according to the McFarland standard of 0.5 (Rolim et al., 2019) concentration for each of the microorganisms grown from the plates there in solid form.

Muller Hinton broth for bacteria, Roswell Park Memorial Institute (RPMI) broth for yeast, and solutions containing different concentrations of AgNPs were added to 96-well microplates. Firstly, wells were designed and then a series of dilutions were performed. After the microorganism suspension prepared for each strain was added to wells, the same procedures were repeated for vancomycin (used for Gram-positive strains), colistin (used for Gram-negative strains), and fluconazole (used for *C*. *Albicans* yeast) antibiotics to compare the inhibitory effects of AgNPs.

The microplates were incubated to propagate at 37°C for 24 hours. At the end of this period, the well before the well where propagation started was determined as the minimum inhibition concentration (MIC).

### 2.5. Examining the Cytotoxic Activities of AgNPs via the MTT Assay

Glioblastoma (U118), human colorectal adenocarcinoma (Caco-2), and ovarian sarcoma (SKOV-3) cell lines were commercially purchased from the American Type Culture Collection (ATCC). Cytotoxic activity applications on these cells were carried out at the Cell Culture Laboratory of Dicle University's Scientific Research Centre.

U118 and Caco-2 cells used were cultured in 75 t-flasks with Dulbecco's Modified Eagle's Medium (DMEM). Skov-3 cells were cultured in 75 t-flasks with the Roswell Park Memorial Institute (RPMI) 1640 medium. The cultured flasks were incubated at 37°C, under 5% CO_2_, 95% air, and humidity conditions. After the cells reached approximately 80% confluency, the cell was counted by using a hemocytometer and 10^4^ cells were seeded per well of 96-well plates and subjected to overnight incubation. After the incubation period, the cells were treated with nanoparticles in concentrations of 200 *μ*g/mL, 100 *μ*g/mL, 50 *μ*g/mL, and 25 *μ*g/mL and incubated for 48 hours. After this period of waiting, the MTT solution was added to the plate wells, and 3 hours after incubation with MTT reagent, the medium was aspirated gently and 100 *μ*l of DMSO was added to each well and incubated for 15 min at RT with gentle shaking. The absorbance of the microplates at 540 nm wavelength was measured using the Multi ScanGo, Thermo device.

Utilizing these absorbance values, the concentration in which the percentage of the viability of AgNPs is inhibited on cells was calculated.

% viability = *U*/*C* *∗* 100 [25, 26], where *U* is the absorbance of cells treated with AgNPs and *C* defines the absorbance values of control cells.

### 2.6. Statistical Analysis

The experiments were performed in triplicate by means of the *t*-test and ANOVA. *P* < 0.05 was regarded as significant.

## 3. Results and Discussion

### 3.1. UV-Vis Spectrophotometer Data

Colour transformation from yellow to dark brown was observed one hour after mixing the plant extract and the 10 mM AgNO_3_ solution [8]. This color change is caused by the reduction of silver ions to AgNPs and the occurrence of vibrations (SPR) on the plasma surface [6]. The maximum absorbance was found to be at 463 nm after analyzing the samples taken periodically via the UV-Vis device (Figure 1). Colour transformation and maximum absorbance data show that AgNPs formed in the reaction liquid [27]. In the synthesis study with *Holoptelea integrifolia* plant extract, 460 nm maximum absorbance data were evaluated with the presence of AgNPs [18]. In another synthesis study of plant origin, 460 nm was associated with the formation and presence of AgNPs [28].

### 3.2. FTIR Data

FTIR data were evaluated to examine the functional groups involved in the formation of AgNPs. The frequency shifts that occurred between 3334.96 and 3338.80 cm^−1^ and 1635.35 and 1634.97 cm^−1^ occurred, suggesting that the functional groups of–OH (hydroxyl) [29] and C=O (I amide) [30], respectively, play a role in the reduction (Figure 2).

### 3.3. XRD Data

The X-ray diffraction values of the peaks (111), (200), (220), and (311) at 2*θ* were found to be 38.14, 44.09, 64.44, and 77.40, respectively (Figure 3). Based on these values, the crystal structure was determined to be cubic, and the crystal nanosize was calculated as 11.61 nm using the Debye–Scherrer equation (*D* = *Kλ*/(*β* cos*θ*)) [31]. The meanings of the symbols in this equation are as follows: *D* = particle size, *K*: constant value (0.90), X-ray wavelength *λ* value: 1.5418 Å, *β*: value of the peak at the maximum height (FWHM), and Bragg *θ*: angle of a high peak. In some studies, the crystal nanosize of AgNPs 14.58 nm [32], 12.63 nm [33], and 2.18 nm was calculated using the Debye–Scherrer equation [34].

### 3.4. FESEM, TEM, and EDX Data

FESEM, TEM, and EDX analysis data were used to determine the morphological structures and element compositions of AgNPs. FESEM and TEM images showed that the AgNPs obtained were spherical, and the presence of substantially strong silver peaks [18] were detected in the EDX profile. Weak peaks in the EDX profile such as Cl, O, and C were due to phytochemicals in the extract [35] (Figure 4).

### 3.5. Evaluation of Antimicrobial Activities of AgNPs

Metallic silver ions are inert in their dry state. They show highly reactive properties when they are ionized in water. Ionized silver contacts microorganisms via its electrostatic attraction force. This causes an increase in reactive oxygen species (ROS). The structure of the cell wall is disrupted by the increase in ROS. The structure of the cell membrane and nucleus membrane also deteriorates. Structures such as DNA and RNA have a high affinity for these species. By affecting the activities of these structures, they disrupt their functions and cause cell destruction and death [3, 36].

Antimicrobial effects of AgNPs were tested on pathogens such as Gram-positive and Gram-negative bacteria and yeast. The inhibitive effects of silver nitrate, AgNPs, and standard antibiotics on tested microorganisms were compared. Based on these results, the AgNPs were found to be effective at least 2 more times than the antibiotics used in the treatment (Table 1).

AgNPs obtained with *Pistacia terebinthus* extract were said to be effective on *S*. *aureus*, *E*. *coli*, and *C*. *albicans* microorganisms at concentrations of 0.04, 0.66, and 0.16 *μ*g/mL, respectively [31, 33]. In a study where different sizes were synthesized, the MIC concentrations of AgNPs that were 5 nm in size for *B*. *subtilis*, *S*. *aureus*, and *E*. *coli* were reported in size 0.8, 6, and 6 *μ*g/mL, respectively [37]. In another similar study, a concentration of 30 *μ*g/mL was effective for *Pseudomonas aeruginosa* ATCC 27853 [35]. In another study, it was reported that silver nanoparticles showed effective inhibition of the growth of Gram-negative and Gram-positive bacteria [24, 38].

### 3.6. Investigation of Cytotoxic Activities of AgNPs

The cytotoxic activities of AgNPs synthesized using *Ananas comosus* peel extract on U118, CaCo-2, and Skov-3, cancer cells were examined via the MTT method (Table 2). According to the data obtained, on CaCo-2 cell lines at a concentration of 25 *μ*g/mL, it showed an inhibitory effect of 81% depending on the % viability of 18.20 on the cell line. Increases in the percentage of viability in some cell lines during transitions to high concentrations were due to the proliferative features of cancer cells [39].

AgNPs show a strong oxidative structure. Ag^+^ release can induce cytotoxic and genotoxic formations in biological structures, and it is important to evaluate these effects [40].

AgNPs interact with the cell surface and cause the cellular composition to deteriorate [12]. AgNPs settle in structures such as the cell membranes, nucleus, and mitochondria. AgNPs cause an increase in ROS; besides, they show toxic effects by stimulating apoptosis [39, 41].

In a study conducted to examine the toxic effects of AgNPs, a concentration of 3.75 *μ*g/mL showed toxic effects on Caco-2 cells [42]. In another study, the concentration at which it showed toxic effects on Skov-3 cells was determined to be 9.4 *μ*g/mL [43].

Some features can have a significant effect on the toxicity of nanoparticles. Concentration, exposure time, burden, the chemistry of surface composition, degree of accumulation, shape, and size are some of these [3, 23].

The different cytotoxic concentrations of AgNPs in the studies may be due to the synthesis of AgNPs from different sources or their different sizes and morphological structures.

## 4. Conclusions

Antibiotic resistance is a serious problem. AgNPs will significantly contribute to the research for antimicrobial agents to solve this situation. Studies have demonstrated that AgNPs synthesized with biological sources show biocompatible properties.

AgNPs are effective on pathogenic species in many studies. However, the toxic effects of their use should also be noted. Cytotoxic activity studies are significant data that will help eliminate this concern.

Waste is among the ever-growing problems in our world. A wide variety of methods are being developed to use such waste in the fields and areas that will benefit people.

In the study, AgNPs were synthesized in an easy, economical, and ecofriendly method by using the bioactive components in pineapple fruit peels to reevaluate waste. The obtained AgNPs were characterized via UV-Vis, FTIR, XRD, TEM, FESEM, and EDX data in which they exhibited at 463 nm maximum absorbance, 11.61 nm in crystal nanosize, and spherical appearance. The AgNPs showed antimicrobial effects at low concentrations. To examine the usability of these particles as an anticancer agent, their cytotoxic effects were examined, and it was determined that 25 *μ*g/mL concentration showed 25–81% inhibition in different cancer cell lines. In addition, the anticancer effect of AgNPs obtained by green synthesis on the U118 cancer cell line was investigated for the first time in this study. The resulting AgNPs can be developed and used in the medical and pharmaceutical industries.

## Figures and Tables

**Figure 1:** UV-Vis showing the formation and presence of AgNP spectrophotometer data.

**Figure 2:** Evaluation of functional groups that play a role in the reduction in plant extract with FTIR spectral analysis data. (a) *Ananas comosus* fruit peels; (b) green synthesized AgNP pattern.

**Figure 3:** X-ray diffraction (XRD) patterns of AgNPs.

**Figure 4:** FESEM (a), TEM (b), and EDX (c) analysis data of silver nanoparticles.

**Table 1:** MIC values of AgNPs, silver nitrate solution (5 mM AgNO_3_), and effect of standard antibiotics on the growth of pathogen bacterial and fungal species.

Pathogen microorganism	AgNPs (*μ*g/mL)	Silver nitrate (*μ*g/mL)	Standard antibiotics^*∗*^*(μ*g/mL)
*S*. *aureus ATCC 29213*	0.50	2.65	2.00
*B*. *subtilis ATCC 11774*	0.25	1.32	1.00
*E*. *coli ATCC 25922*	1.00	0.66	2.00
*P*. *aeruginosa ATCC27833*	2.00	1.32	4.00
*C*. *albicans* (*clinical isolate*)	0.50	0.66	2.00

^*∗*^Vancomycin: Gram-positive strains (*S*. *aureus* and *B*. *subtilis*), colistin: Gram-negative strains (*E*. *coli* and *P*. *aeruginosa*), and fluconazole: *C*. *albicans*.

**Table 2:** Cytotoxic effects of AgNPs on cell lines (*n* = 3, mean ± standard deviation).

	Cell lines	25 (*μ*g/mL)	50 (*μ*g/mL)	100 (*μ*g/mL)	200 (*μ*g/mL)
% viability	U118	74.90 ± 0.001^a^	71.57 ± 0.001	66.93 ± 0.003	17.00 ± 0.001
	CaCo-2	18.20 ± 0.002	9.42 ± 0.002	9.62 ± 0.001	12.51 ± 0.001
	Skov-3	57.92 ± 0.002	55.34 ± 0.001	45.88 ± 0.002	19.78 ± 0.002

^a^Standard deviation.

## Data Availability

All data used to support the findings of this study are included in the article.
